# Eye Movement Signal Classification for Developing Human-Computer Interface Using Electrooculogram

**DOI:** 10.1155/2021/7901310

**Published:** 2021-12-08

**Authors:** M. Thilagaraj, B. Dwarakanath, S. Ramkumar, K. Karthikeyan, A. Prabhu, Gurusamy Saravanakumar, M. Pallikonda Rajasekaran, N. Arunkumar

**Affiliations:** ^1^Department of Electronics and Instrumentation Engineering, Karpagam College of Engineering, Coimbatore, Tamil Nadu, India; ^2^Department of Information Technology, SRM Institute of Science and Technology, Chennai, Tamil Nadu, India; ^3^School of Computing, Kalasalingam Academy of Research and Education, Krishnankoil, Virudhunagar, Tamil Nadu, India; ^4^Department of Electrical and Electronics Engineering, Ramco Institute of Technology, Rajapalayam, Tamil Nadu, India; ^5^K. Ramakrishnan College of Engineering, Trichy, Tamil Nadu, India; ^6^Department of Electrical and Electronics Technology, Ethiopian Technical University, Addis Ababa, Ethiopia; ^7^Department of Electronics and Communication Engineering, Kalasalingam Academy of Research and Education, Krishnankoil, Virudhunagar, Tamil Nadu, India; ^8^Department of Biomedical Engineering, Rathinam Technical Campus, Coimbatore, Tamil Nadu, India

## Abstract

Human-computer interfaces (HCI) allow people to control electronic devices, such as computers, mouses, wheelchairs, and keyboards, by bypassing the biochannel without using motor nervous system signals. These signals permit communication between people and electronic-controllable devices. This communication is due to HCI, which facilitates lives of paralyzed patients who do not have any problems with their cognitive functioning. The major plan of this study is to test out the feasibility of nine states of HCI by using modern techniques to overcome the problem faced by the paralyzed. Analog Digital Instrument T26 with a five-electrode system was used in this method. Voluntarily twenty subjects participated in this study. The extracted signals were preprocessed by applying notch filter with a range of 50 Hz to remove the external interferences; the features were extracted by applying convolution theorem. Afterwards, extracted features were classified using Elman and distributed time delay neural network. Average classification accuracy with 90.82% and 90.56% was achieved using two network models. The accuracy of the classifier was analyzed by single-trial analysis and performances of the classifier were observed using bit transfer rate (BTR) for twenty subjects to check the feasibility of designing the HCI. The achieved results showed that the ERNN model has a greater potential to classify, identify, and recognize the EOG signal compared with distributed time delay network for most of the subjects. The control signal generated by classifiers was applied as control signals to navigate the assistive devices such as mouse, keyboard, and wheelchair activities for disabled people.

## 1. Introduction

Healthy human beings use their muscles to move, drive vehicles, and move objects. The muscles receive commands from the brain. Certain neuromuscular disorders impair the communication between the brain and the muscles, causing partial or total paralysis depending on the severity of disorders. In most cases, eye muscle functions are not initially affected. These disorders do not impair cognitive abilities, and such individuals are aware of their environment, creating a locked-in state. Medical research helps such individuals live longer, and hence rehabilitation becomes essential to improve their lifestyle and reduce the burden on their caregivers. The human-computer interface provides a digital communication channel for paralyzed people by assisting human cognitive or motor neuron function through bypassing the biological channel communication. Some of the prominent interfaces developed for impaired persons include smartphones, keyboards, game controllers, sleep monitoring systems, and drowsiness detection systems [1–12].

Electrooculography (EOG) principle was used widely and successfully to detect eye movements to control the human-computer interface because of its noninvasive, portable, and inexpensive activities and because it can be used in almost all environments [13]. In recent years, much research relating to electrooculography supported interface for HCI has been matured to overcome the problem that occurred due to the locked-in state and motor neuron disease. In most of the previous studies, eye blink was defined as an election command for completing the tasks, but sometimes the subject or person was unable to control the eye blinks because blinks would occur unwillingly. To avoid this condition, this paper establishes a new protocol for acquiring signals for both events and nonevents to ensure the possibilities of nine states of HCI by using different eleven eye movements. From these eleven different eye movements, eight were considered as events and three were nonevents. Eye blinks, open, and stare were considered the nonevents during this study. This research mainly focuses on checking the possibilities of design and developing nine states of HCI using classification techniques and recognition rate of HCI with the help of single-trial analysis and accuracy by using bit transfer rate.

Section 2 provides the background details.  Section 3 explains protocol, preprocessing techniques.  Section 4 details the feature extraction, Section 5 deals with classification techniques used in this investigation. Outcome analysis is presented in Section 6, and the conclusion and future study are discussed in Sections 7 and 8.

## 2. Background Study

Nowadays, electrooculography-based human-computer interaction is used by paralyzed people who have neurodegenerative problems. It acts as a good communication device for conveying their thoughts with others by using the technology. The following are some of the most prominent publications that are useful to people with disabilities: a study by Saravanakumar et al. developed EOG based keyboard system in synchronous mode and asynchronous mode using peak amplitude features and obtained the accuracy of 94.2% and 98.79% [14]. In one of the earliest studies, Barea et al. implemented a wheelchair guidance system, which uses four-state systems to guide a wheelchair to move forward, backward, right, and left. The result obtained in this study shows that weakened individuals frequently involve about 10–15 min to be trained to use this arrangement [15]. Thilagaraj et al. devised the assistive device for ALS and semiparalyzed persons using spectral density features with a dynamic network model from twenty individuals and obtained the accuracy of 91.95% and 90.28 [16]. Another study by Tsai et al. concentrated on an eye writing system using EOG signals of eye movements corresponding to pattern recognition of ten Arabic numerals and four mathematical operators and attained 95% accuracy compared to other writing systems [17]. He and Li modeled the audio speller for LIS person through EOG signals using waveform detection algorithm and SVM algorithm and obtained an accuracy of 94.40% [18].

Jayaprbhu et al. developed aided assistive intelligence system for ALS persons using RMS features trained with PNN architecture models from 15 subjects and obtained an accuracy of 94.00% for young aged subjects, 93.27% for old aged subjects, and 90.37% for ALS-affected individuals [19]. Supratak et al. created a sleep detection system for drivers using time-invariant features with the CNN network model and obtained the accuracy of 86.20% and 73.70% for two different datasets [20]. Obeidat et al. developed a wheelchair for a paralyzed person using Bayesian Linear Discriminant Analysis and obtained an accuracy of 95% from fourteen subjects [21]. Jayaprbhu et al. developed EEG-based BCI for ALS-affected persons using the convolution neural network and cross power spectral density for four subjects from fifteen subjects and obtained the accuracy of 91.18% and 86.88% [22]. Xiao et al. modeled four-state EEG-based BCI for SCI-affected individuals using CWT featured with a hybrid neural network and obtained an accuracy of 93.86% [23]. Kai et al. designed the rehabilitative device for LIS patients using local binary patterns features with Grey Wolf optimization algorithm and obtained 98.33% to 88.33% for the subject's age group between 20 and 60 from nine subjects [24].

Dev et al. designed a wheelchair controller for quadriplegic patients using PSD features and a fuzzy classifier and obtained good accuracy using one electrode system from NeuroSky Headset [25]. Lokman et al. created BCI to control the finger movement from thirteen subjects using genetic algorithm features with MLP and SVM classifiers and obtained the accuracy of 97.34% and 97.46% [26]. Turnip et al. modeled wheelchairs for SCI-affected individuals for four tasks and obtained 90% accuracy using ANFIS classifiers from four subjects belonging to the age group between 25 and 26 [27]. Ilyas et al. developed BCI to determine the patterns using several classifiers and obtained the maximum accuracy of 73.03% for logistic regression and 68.97% for SVM classifiers [28]. A background study on EOG classification exposed that very limited work has been presented on identifying the EOG signals using Elman and Distributed time delay neural network, and much research focuses on conventional movements only. Through this research, we consider the possibility of recognizing eight-task (events) and three-task (nonevents) movements using feedback networks. The achievement of the feature extraction approach was compared using a feedback network to confirm the outcomes.

## 3. Experimental Protocol

We started our study with a preliminary study with two subjects, a male and a female, to determine the signals patterns. For each individual subject, the pattern generation was different, and also we identified that all the different tasks produced different patterns. Therefore, we concluded that classifying all the tasks was possible during the study.

ADT26 bioamplifier was used to gather EOG signals for 20 normal persons. Signals gathered from the participants were sampled at 100 HZ and each band was split with 2HZ from 0.1 to 16 Hz. The methodology of the study implemented in this research was described by the same author in his prior study [29, 30].

## 4. Feature Extraction

A feature extraction algorithm using convolution theorem was used to extract the prominent features from the band-pass filtered EOG signals for all eleven tasks. The theorem described that a mathematical operation on two-channel signals *X*_*b*_^*j*^ and *R*_*b*_^*j*^ in time domain equals pointwise multiplication in the frequency domain of the original signals converted. Finally, the convoluted signals F1 and *R*_1_ are written as *F*_1_*∗R*_1_ , so that convolution operator was indicated by using *∗* symbolized:

(1) $$\begin{array}{c} X_{b}^{j}={\left\{\;x_{bi}^{j}\right\}}_{i=1,2,\ldots 100,\;b=1,2,\ldots ,8},\\ R_{b}^{j}={\left\{\;x_{bi}^{j}\right\}}_{i=100,99,\ldots 1,\;b=1,2,\ldots ,8},\\ F_{1}=F\left\{X_{b}^{j}\right\},\\ R_{1}=F\left\{R_{b}^{j}\right\}. \end{array}$$

Let F represent the Fourier transform, so that *F*(*X*_*b*_^*j*^) is a Fourier signal and *F*(*R*_*b*_^*j*^) is a reverse and shifted Fourier signal of the Fourier transform of F_1_ and R_1_ correspondingly. Then,

(2) $$\begin{array}{c} F\left\{F_{1}*R_{1}\right\}=F\left\{F_{1}\right\}\cdot F\left\{R_{1}\right\}, \end{array}$$

where the dot indicates the pointwise multiplication. Thus, equation (2) can also be written as

(3) $$\begin{array}{c} F\left\{F_{1}\cdot R_{1}\right\}=F\left\{F_{1}\right\}*F\left\{R_{1}\right\}. \end{array}$$

By implementing the convolution equation, we can write down

(4) $$\begin{array}{c} F_{1}*R_{1}=\sum_{n=0}^{N-1}\left\{F\left\{F1\right\}.F\left\{R1\right\}\right\}. \end{array}$$

From this feature extraction technique, 16 features were taken out for individual trial. The features were extracted for 10 such trials for each task. A neural network classifier was implemented to train and test 110 data samples for one subject. The feature sets obtained from the single trial for each task are demonstrated in Figure 1.

## 5. Classification Techniques

To categorize the signal obtained from the eye movements for 20 subjects, two neural network models were planned to recognize the eleven different tasks. Two classical networks, particularly the ERNN and DTDNN, were applied in this study. The convolution features were given as input to the following networks. Outcomes of two network models were related to validating the possibility of designing multistates HCI.

### 5.1. Elman Recurrent Neural Network (ERNN)

ERNN has feedback connections that affix the capability to study the physical aspects of the data. The network architecture consists of a context layer, which was equal to the hidden layer in an ordinary network model to make a copy. The main aspects of this layer maintain the previous state of the hidden layer at the previous pattern arrangement. Due to this reason, the training time testing time and classification rate of the network model were higher than those of FFNN [31–34].

### 5.2. Distributed Time Delay Neural Network

A DTDNN was one of the most powerful dynamic network models, and its performance was high compared to other static network models because it has a capacity to learn time varying and also the sequential patterns due to its memory storage. The layers involved in this architecture have biases, so each layer has added the weight from the earlier layers, and the last layer was completed with output layers. It assigns the tapped delay lines throughout the network. The only difference between the DTDNN and the TDNN is that the second input argument is a cell array that contains the tapped delay to be used in each layer. It was similar to FFNN, except that each input and layer weight have a tap delay line associated with it [35–38].

During the parameters settings, we fixed the neural network classifier in the below-mentioned condition. The two network models were trained using backpropagation (Gradient Descent) for the ERNN model and Levenberg backpropagation training algorithm for the DTDNN model with eight hidden neurons, sixteen input neurons, and four output neurons. The two network models were trained with 100% data samples and trained with 75% for each individual subject, and also, we fixed testing error tolerance of 0.1 during the testing with a .001 learning rate of the network model experimentally. During the classification, we normalized the samples between zero and one using the normalization procedure. The maximum iteration of the network was fixed and limited to 1000, and network error falls below 0.001 to determine the network performance [34, 39, 40]. Figures 2 and 3 present the construction of the ERNN and DTDNN models used in this experiment.

## 6. Outcome Analysis

Tables 1 and 2 showed the average accuracy of the network models implemented in the study. The results showed that the ERNN model has the highest overall classification accuracy of 90.82%, whereas the DTDNN model has the highest overall classification accuracy of 90.56%. The maximum classification accuracy of 91.91% and 91.76% was observed for subject 12. The average maximum classification accuracy of 93.97% and 3.87% was observed. The average minimum classification accuracy of 86.10% and 86.06% was observed. Average testing and training times for twenty subjects were 5.35 and 0.9205 seconds and 3.64 and 0.6545 for the convolution features using ERNN and DTDNN, respectively. From the study, we observed that the ERNN model performed better than the DTDNN model throughout the investigation, which is depicted in Figure 4. From the outcomes obtained in recognizing the eleven eye movements, it was seen that the performance of ERNN models using convolution features was high compared to the DTDNN architecture used in this study.

### 6.1. Single-Trial Analysis (STR) Using ERNN and DTDNN with Convolution Features

From the STR, it was concluded that S1 achieved 80% accuracy for rapid movement and open and 70% accuracy for left, up right, down right, up left, down left, close, and stare. S2 achieved 80% accuracy for up right, up left, and close and 70% accuracy for right, left, down right, down left, and stare. S3 achieved 80% accuracy for left, down right, and stare and 70% accuracy for up right, down left, and open. S4 achieved only 80% accuracy for down right, down left, open, and stare and 70% accuracy for right, up right, up left, and close. S5 achieved only 80% accuracy for down right and 70% accuracy for left, up right, up left, open, and stare. S6 achieved only 80% accuracy for left and down right and 70% accuracy for up right, up left, and down left. S7 achieved only 80% accuracy for left, down right, and up left and 70% accuracy for right, up right, and stare. S8 achieved 100% accuracy for close; 90% accuracy for left; 80% accuracy for up right, up left, and down left; and 70% accuracy for right, down right, open, and stare. S9 achieved 80% accuracy for down right and 70% accuracy for left, up left, and open. S10 achieved 100% accuracy for left and 80% accuracy for up right and stare. S11 achieved 80% accuracy for lateral movement and close and 70% accuracy for up right, open, and stare. S12 achieved 80% accuracy for open and stare and 70% accuracy for left, up right, down right, up left, and down left. S13 achieved 80% accuracy for down right and 70% accuracy for down left and stare. S14 achieved 80% accuracy for up right and 70% accuracy for left, up left, and stare. S15 achieved only 80% accuracy for up left and 70% accuracy for up right, down right, and down left. S16 achieved 80% accuracy for down left and open and 70% accuracy for left, up right, and stare. S17 achieved 80% accuracy for up right and down left and 70% accuracy for open and stare. S18 achieved 90% accuracy for open, 80% accuracy for left up right and stare, and 70% accuracy for up left. S19 achieved 80% accuracy for down right and 70% accuracy for left, up right, open, and stare. S20 achieved 80% accuracy for up right and stare and 70% accuracy for left and open using the ERNN model.

From the STR, it was concluded that S1 achieved 80% accuracy for rapid movement and open and 70% accuracy for left, up right, down right, up left, down left, close, and stare. S2 achieved 80% accuracy for up right, up left, and close and 70% accuracy for right, left, down right, down left, and stare. S3 achieved 80% accuracy for left, down right, and stare and 70% accuracy for up right, down left, and open. S4 achieved only 80% accuracy for down right, down left, open, and stare and 70% accuracy for right, up right, up left, and close. S5 achieved only 70% accuracy for left, up right, up left, open, and stare. S6 achieved only 80% accuracy for left and down right and 70% accuracy for up right, up left, and down left. S7 achieved only 80% accuracy for left, down right, and up left and 70% accuracy for right, up right, and stare. S8 achieved 100% accuracy for close; 90% accuracy for left; 80% accuracy for up right, up left, and down left; and 70% accuracy for right, down right, open, and stare. S9 achieved 80% accuracy for down right and 70% accuracy for left, up left, open, and stare. S10 achieved 100% accuracy for left; 80% accuracy for up right and stare; and 70% accuracy for up left, open, and stare. S11 achieved 80% accuracy for lateral movement and close and 70% accuracy for up right, open, and stare. S12 achieved 80% accuracy for open and close and 70% accuracy for left, up right, down right, up left, and down left. S13 achieved 80% accuracy for down right and 70% accuracy down left and stare. S14 achieved 80% accuracy for up right and 70% accuracy for left, up left, and stare. S15 achieved only 80% accuracy for up left and 70% accuracy for up right, down right, and down left. S16 achieved 80% accuracy for down left and open and 70% accuracy for left, up right, and stare. S17 achieved 80% accuracy for up right and down left and 70% accuracy for open and stare. S18 achieved 90% accuracy for open, 80% accuracy for left up right and stare, and 70% accuracy for up left. S19 achieved 80% accuracy for down right and 70% accuracy for left, up right, open, and stare. S20 achieved 80% accuracy for up right and stare and 70% accuracy for left and open using the DTDNN model.

The result of the nine-state HCI system designed for each subject was explored through a single-trial analysis using ERNN and DTDNN for convolution features. From the STR, it was observed that, for subjects 7 and 8, the accuracy rate was high at a mean of 90% for events and 85% for nonevents using convolution features, and for subject 13, the acceptance rate was low at a mean of 70% for events and 75% for nonevents using convolution features with ERNN and DTDNN network model used in this investigation. From the single-trial analysis, it was evident that eighty percentages of the signals have a recognition rate of eight and above for some subjects such as S1, S2, S3, S4, S5, S13, S19, and S20 where the recognition rates were not appreciable. From the analysis, we concluded that more training was required to improve the recognition accuracy of the events as well as nonevents. From the result, it was identified that practicability of developing a nine-state HCI is possible for some subjects participating in this experiment using convolution features for DTDNN, while for some of the subjects such as S1, S2, S3, S4, S5, S13, S19, and S20, the mean recognition accuracy of nine-state HCI was around 80% only, so the subjects involved in the study were not able to perform some of the trials correctly and feel that the task was hard to perform continuously. They were also unable to switch over from one task to another immediately.

Sensitivity and specificity were the mathematical evaluation of the classification test, where sensitivity calculates the events that were correctly identified. The sensitivity, specificity, and accuracy of the individual subject were calculated from equations (5), (6), and (7):

  True positive (TP) = correctly classified trials
  False positive (FP) = incorrectly classified trials
  True negative (TN) = correctly classified nonevent trials
  False negative (FN) = incorrectly classified nonevents trials

(5) $$\begin{array}{c} \text{Sensitivity}=\frac{\text{TP}}{\left(\text{TP}+\text{FN}\right)}. \end{array}$$

Specificity calculates the events that were identified as wrongly classified:

(6) $$\begin{array}{c} \text{Specificity}=\frac{\text{TN}}{\left(\text{TN}+\text{FP}\right)}. \end{array}$$

### 6.2. Accuracy

The accuracy of the subject was measured by differentiating events and nonevents cases correctly. To calculate the accuracy test, estimate the proportion of TP and TN in all appraised cases proposed by [41, 42]. The mathematical formula to calculate the accuracy is stated as

(7) $$\begin{array}{c} \text{Accuracy}=\frac{\left(\text{TP}+\text{TN}\right)}{\left(\text{TP}+\text{TN}+\text{FP}+\text{FN}\right)}. \end{array}$$

From the investigational result, it was analyzed that the convolution features using ERNN outperform the DTDNN model for some subjects. At the same time, the DTDNN model gave better accuracy for some subjects during this study. This confirms that EOG signals were subject variants. After comparison, it was analyzed that ERNN with convolution features was analyzed to be the best classifier model among the other network model designed for eleven tasks. The individual recognizing accuracy of subjects was determined using the GUI designed using MATLAB demonstrated in Figure 5.

### 6.3. Evaluation of Bit Transfer Rate (BTR)

The HCI performance can also be evaluated using the BTR. BTR states the number of bits transmitting per unit of time. This criterion includes accuracy and speed in a single value. The BTR for the eleven tasks using convolution features for ERNN and DTDNN are shown in Tables 3 and 4. The bit transfer rates have been determined from the following:

(8) $$\begin{array}{c} \text{Bit transfer rate}=\frac{60}{T_{\text{act}}}\left[\log_{2}\;n+p_{a}\log_{2}p_{a}+\left(1-p_{a}\right)\log_{2}\frac{1-p_{a}}{n-1}\right]. \end{array}$$

*n* indicates the number of eye movements, *T*_act_ represents action period, *p*_*a*_ specifies the mean accuracy, and 1 −  *p*_*a*_ shows mean recognition error [42, 43].

#### 6.3.1. Bit Transfer Rate for Convolution Features Using ERNN

The results of the BTR for an individual subject are shown in Table 3 for ERNN using convolution features. Single-trial analysis results of the classifier show that the ERNN has a maximum accuracy for subject 7 and minimum accuracy for subject 13 using single-trial EOG classification for convolution features. The maximum bit rate for the ERNN using convolution features of 83.55% was obtained for S12 and the minimum bit rate for the ERNN using convolution features of 80.34% with samples from ten trials which is shown in Figure 6.

#### 6.3.2. Bit Transfer Rate for Convolution Features Using DTDNN

The results of the BTR for an individual subject are shown in Table 4 for DTDNN using convolution features. Single-trial analysis results of the classifier show that the DTDNN has a maximum accuracy for subject 8 and minimum accuracy for subject 13 using single-trial EOG classification for convolution features. The maximum bit rate for the DTDNN using convolution features of 83.24% was obtained for S12 and the minimum bit rate for the DTDNN using convolution features of 79.98% with samples from ten trials which is shown in Figure 7.

The accuracy of both network models was correlated based on their accuracy and performance. From the analysis, the ERNN model was significantly higher when related to that of the DTDNN model. From the results, we finally concluded that designing nine-state HCI is possible by using ERNN model with convolution features.

#### 6.3.3. Limitation of the Study

The system was especially designed for patients with eye movement's activities. The patients without eye movement activities were unable to use this system.

## 7. Conclusion

Eleven tasks were requested to be executed by each individual subject using the ADI T26 Bioamplifier. Two new movements were projected in this research. A new feature extraction algorithm using the convolution theorem has been implemented for extracting features. From the results, it was finalized that the network model using the Elman Recurrent Network model with convolution features was more appropriate for recognizing all the eleven eye movements with the recognizing performance of 90.82%. Single-trial analysis was conducted for an individual subject to analyze the performance of individual subjects. The results show that eye movement classification was subject-oriented. From the bit transfer rate, it was analyzed that the classification performance of convolution features using ERNN was better compared to the DTDNN network model. The experimental analysis proved that the ERNN models were more appropriate for categorizing the collected signals for eleven tasks (both events and nonevents) using convolution features.

## 8. Future Study

Our future extension of this study is to realize online human-machine interaction for nine-state HCI to recognize the high-level human activity in a more efficient way for severely paralyzed persons to fully fill their needs without others' help.

## Figures and Tables

**Figure 1:** Signals extracted by implementing the feature extraction technique for (a) right, (b) left, (c) up right, (d) down right, (e) up left, (f) down left, (g) rapid movement, (h) lateral movement, (i) open, (j) close, and (k) stare tasks for Subject 2 using convolution theorem.

**Figure 2:** Elman recurrent neural network model.

**Figure 3:** Distributed time delay neural network model.

**Figure 4:** Average classification accuracy of the convolution features using ERNN and DTDNN.

**Figure 5:** Recognizing accuracy evaluation using GUI.

**Figure 6:** Maximum, minimum, and mean accuracy and bit transfer rate for convolution features using ERNN.

**Figure 7:** Maximum, minimum, and mean accuracy and bit transfer rate for convolution features using DTDNN.

**Table 1:** Performance accuracy of convolution features using ERNN.

S. no.	Sub.	Hidden neuron	Training time (sec)	Testing time (sec)	Recognizing accuracy			
					Max	Min	Mean	Std.
1	S1	8	5.31	0.92	93.64	83.64	90.73	2.60
2	S2	8	5.12	0.94	93.64	87.27	90.86	2.03
3	S3	8	5.38	0.91	94.55	85.45	90.94	2.46
4	S4	8	5.43	0.88	93.64	86.36	90.90	2.13
5	S5	8	5.42	0.93	93.78	85.45	90.58	2.32
6	S6	8	5.45	0.84	93.64	86.36	90.59	2.23
7	S7	8	5.43	0.94	93.64	85.56	90.77	2.48
8	S8	8	5.32	0.92	93.64	86.36	90.90	2.22
9	S9	8	5.34	0.86	94.55	85.45	90.91	2.15
10	S10	8	5.30	0.89	93.64	84.55	90.31	2.41
11	S11	8	5.32	0.96	93.64	86.36	90.58	2.17
12	S12	8	5.41	0.93	95.55	88.18	91.91	2.04
13	S13	8	5.39	0.95	93.64	86.36	90.90	1.93
14	S14	8	5.34	0.92	93.64	86.36	91.12	2.12
15	S15	8	5.34	0.95	94.55	87.09	90.71	1.92
16	S16	8	5.43	0.89	94.55	85.56	90.77	2.20
17	S17	8	5.52	0.90	93.64	86.36	90.68	2.00
18	S18	8	5.42	0.92	93.64	85.56	90.77	2.22
19	S19	8	5.42	0.97	93.64	87.27	90.82	2.09
20	S20	8	5.40	0.99	94.55	86.36	90.64	1.94

**Table 2:** Performance accuracy of convolution features using DTDNN.

S. no.	Sub.	Hidden neuron	Mean training time (sec)	Mean testing time (sec)	Recognizing accuracy			
					Max	Min	Mean	Std.
1	S1	8	3.51	0.67	93.64	86.36	90.41	2.14
2	S2	8	3.56	0.61	93.72	85.56	90.49	1.88
3	S3	8	3.57	0.63	93.74	86.36	90.40	2.25
4	S4	8	3.70	0.65	92.74	86.36	90.58	1.79
5	S5	8	3.48	0.62	93.64	85.45	90.32	2.83
6	S6	8	3.59	0.76	93.64	85.56	90.13	1.99
7	S7	8	3.62	0.62	93.64	85.45	90.59	2.63
8	S8	8	3.62	0.62	93.64	86.36	90.49	1.64
9	S9	8	3.72	0.65	93.64	85.45	90.34	2.00
10	S10	8	3.59	0.63	93.64	86.36	90.23	2.31
11	S11	8	3.44	0.61	94.55	85.56	90.47	2.23
12	S12	8	3.55	0.63	94.55	88.18	91.76	1.79
13	S13	8	3.71	0.63	94.55	86.36	90.63	2.13
14	S14	8	3.92	0.61	94.55	85.45	90.86	2.26
15	S15	8	3.68	0.63	93.64	86.36	90.50	1.97
16	S16	8	3.60	0.63	94.55	85.55	90.59	2.08
17	S17	8	3.82	0.73	93.64	86.36	90.54	1.87
18	S18	8	3.65	0.70	93.64	86.36	90.59	2.17
19	S19	8	3.67	0.73	93.64	85.45	90.58	1.79
20	S20	8	3.84	0.73	94.55	86.36	90.73	2.50

**Table 3:** Bit transfer rate of ERNN using convolution features.

S. no.	Sub.	Bit transfer rate			
		Maximum accuracy	Minimum accuracy	Mean accuracy	BTR accuracy
1	S1	93.64	83.64	90.73	81.17
2	S2	93.64	87.27	90.86	81.43
3	S3	94.55	85.45	90.94	81.59
4	S4	93.64	86.36	90.90	81.51
5	S5	93.78	85.45	90.58	80.87
6	S6	93.64	86.36	90.59	80.89
7	S7	93.64	85.56	90.77	81.25
8	S8	93.64	86.36	90.90	81.51
9	S9	94.55	85.45	90.91	81.53
10	S10	93.64	84.55	90.31	80.34
11	S11	93.64	86.36	90.58	80.87
12	S12	95.55	88.18	91.91	83.55
13	S13	93.64	86.36	90.90	81.51
14	S14	93.64	86.36	91.12	81.95
15	S15	94.55	87.09	90.71	81.13
16	S16	94.55	85.56	90.77	81.25
17	S17	93.64	86.36	90.68	81.07
18	S18	93.64	85.56	90.77	81.25
19	S19	93.64	87.27	90.82	81.35
20	S20	94.55	86.36	90.64	80.99

**Table 4:** Bit transfer rate of DTDNN using convolution features.

S. no.	Sub.	Bit transfer rate			
		Maximum accuracy	Minimum accuracy	Mean accuracy	BTR accuracy
1	S1	93.64	86.36	90.41	80.53
2	S2	93.72	85.56	90.49	80.69
3	S3	93.74	86.36	90.40	80.51
4	S4	92.74	86.36	90.58	80.87
5	S5	93.64	85.45	90.32	80.36
6	S6	93.64	85.56	90.13	79.98
7	S7	93.64	85.45	90.59	80.89
8	S8	93.64	86.36	90.49	80.69
9	S9	93.64	85.45	90.34	80.39
10	S10	93.64	86.36	90.23	80.18
11	S11	94.55	85.56	90.47	80.65
12	S12	94.55	88.18	91.76	83.24
13	S13	94.55	86.36	90.63	80.97
14	S14	94.55	85.45	90.86	81.42
15	S15	93.64	86.36	90.50	80.71
16	S16	94.55	85.55	90.59	80.89
17	S17	93.64	86.36	90.54	80.79
18	S18	93.64	86.36	90.59	80.89
19	S19	93.64	85.45	90.58	80.87
20	S20	94.55	86.36	90.73	81.16

## Data Availability

The data used to support the findings of this study are available from the corresponding author upon request.
